# Xia-yu-xue decoction (XYXD) reduces carbon tetrachloride (CCl_4_)-induced liver fibrosis through inhibition hepatic stellate cell activation by targeting NF-κB and TGF-β1 signaling pathways

This article has been retracted.

**DOI:** 10.1186/s12906-015-0733-1

**Published:** 2015-06-30

**Authors:** Cheng Liu, Xia Yuan, Le Tao, Zhuoan Cheng, Xiuqin Dai, Xia Sheng, Dongying Xue

**Affiliations:** Experimental Research Center, Putuo Hospital, Shanghai University of Traditional Chinese Medicine, Shanghai, 200062 China; Department of Pharmacy, Putuo Hospital, Shanghai University of Traditional Chinese Medicine, Shanghai, 200062 China; Department of Infectious Disease, Putuo Hospital, Shanghai University of Traditional Chinese Medicine, Shanghai, 200062 China; Department of Pathology, Putuo Hospital, Shanghai University of Traditional Chinese Medicine, Shanghai, 200062 China

**Keywords:** Xia-yu-xue decoction, Hepatic stellate cells, NF-κB, TGF-β1

## Abstract

**Background:**

Hepatic stellate cell (HSC) activation is activated mainly by endotoxin and transforming growth factor (TGF-β1) in chronic liver injury, consequently, can be important therapeutic targets. Xia-yu-xue decoction (XYXD), a classical recipe used in China to treat liver fibrosis, and has been revealed to inhibit hepatic fibrosis in animal models, the mechanism of action of XYXD remains elusive. In the present study, we evaluated whether XYXD reduced endotoxin and pro-fibrogenic pathways induced by lipopolysaccharide (LPS) and TGF-β1 in HSCs.

**Methods:**

The in vivo effect of XYXD on fibrosis progression was assessed in mice model induced by carbon tetrachloride (CCl_4_), The in vitro effect of XYXD on mice GFP-Col-HSC cells was evaluated using LPS and TGF-β1 stimulation.

**Results:**

XYXD treatment reduced CCl_4_-induced liver fibrosis and decreased hepatic hydroxyproline (Hyp) content, the mRNA levels of smooth muscle actin (α-SMA) and Col 1(α1) in fibrotic liver. XYXD suppressed nuclear factor-κB (NF-κB) activation induced by LPS and TGF-β1 assessed by using NF-κB-luciferase reporter. The expression of NF-κB target genes, chemokine (C-C motif) ligand 2 (CCL2) and chemokine (C-X-C motif) ligand 2 (CXCL2) induced by LPS was suppressed after XYXD treatment. The expression of TGF-β1 targets genes, Col1(α1) and tissue inhibitor of metalloproteinases (TIMP1) induced by TGF-β1 was inhibit after XYXD treatment.

**Conclusion:**

XYXD treatment attenuates liver fibrosis by inhibiting HSC activation via inhibition of NF-κB and TGF-β1 signaling pathway, thereby blocking the synthesis of Col1 (α1) and TIMP-1. These findings from present study suggest that XYXD may be a therapeutic decoction for liver fibrosis in which NF-κB and TGF-β1 are thought to take part.

## Background

Liver fibrosis, defined by redundant deposition of extracellular matrix (ECM) and resultant loss of soft and liver function, is the result of wound-healing responses stimulated by various liver injury [1, 2]. In response to liver injury, quiescent hepatic stellate cells (HSCs) are activated and develop a myofibroblast-like phenotype that expresses smooth muscle actin (α-SMA) and profibrogenic genes [3]. HSC activation, the most important event in liver fibrosis, is mediated by many inflammatory and fibrogenic cytokines released from the damaged hepatocytes, circulatory system or from Kupffer cells (KCs). The events subsequent to HSC activation, including the augmented production of collagen, are crucial for the hepatic fibrogenesis cascade. Thus, the HSC activation is an appealing target for the development of new antifibrotic drugs [4, 5].

Xia-yu-xue decoction (XYXD) is a classical recipe from Jin Kui Yao Lue (Synopsis of the Golden Chamber) in 200 AD that has a long history in traditional Chinese medicine. XYXD consists of three medicinal herbs, *Radix et Rhizoma Rhei (10 g), Semen Persicae (10 g), and Eupolyphaga Seu Steleophaga (6 g).* XYXD was used widely in clinical for treatment liver fibrosis patients without side effects [6]. It was reported that XYXD could regulate the balance of MMP2,9/TIMP1,2 in response to LPS stimulation in RAW264.7 cells [7] and inhibit KC activation in pig serum induced liver fibrosis in rats [8]. There was reported that XYXD exerts therapeutic effects by inhibiting HSC activation in carbon tetrachloride (CCl_4_)-induced liver fibrosis in mice [9]. However, scant information is available regarding the antifibrotic mechanism of XYXD action in HSC activation *in vitro* and *in vivo*.

Lipopolysaccharide (LPS) level increased in liver fibrosis from portal and systemic circulation owing to changes in the intestinal mucosal permeability [10]. Toll-like receptor 4 (TLR4) signaling pathway is activated upon LPS stimulation, and induces nuclear factor-κB (NF-κB) activation, which leads to the transcription of inflammatory genes, such as chemokine (C-C motif) ligand 2 (CCL2) and chemokine (C-X-C motif) ligand 2 (CXCL2) in HSCs. We previously showed that LPS stimulation enhanced the response of HSCs to transforming growth factor (TGF-β1) [11]. One the other hand, TGF-β1 derived from injured hepatocytes, activated KCs, increased and bound to TGF receptor in HSCs in chronic liver injury. Thereafter, the downstream signaling such as Smad2/3 phosphorylate, which induce the transcription of pro-fibrogenic genes, such as Col1 (α1) and TIMP1. We hypothesize that XYXD suppresses the LPS-mediated inflammatory signaling through the suppression of NF-κB and TGF-β1-mediated fibrogeinc signaling, thereby attenuating inflammation and profibrogenic response in HSCs.

Consequently, in the present study we applied the CCl_4_ model to examine the anti-fibrotic effects of XYXD in the mice liver. The anti-fibrotic activities were evaluated by histopathology, hepatic hydroxyproline content, and mRNA expression of α-SMA and collagen 1(α1) in vivo. Because the importance of LPS and TGF-β1 in hepatic fibrosis, in vitro we detected the possibility that the anti-fibrotic activities of XYXD might act through the interruption of LPS and TGF-β1 signaling in HSC activation.

## Methods

### Preparation of XYXD

XYXD consists of crude slices were purchased from Shanghai Huayu Chinese Herbs Co Ltd (China) [12] and from the following ratios of three medicinal herbs: *Radix et Rhizoma Rhei* 10 g (2 kg, Cat No:140501), *Semen Persicae* 10 g (2 kg, Cat No:140619), and *Eupolyphaga Seu Steleophaga* 6 g (1.2 kg, Cat No: 141110), total weight 5.2 kg. The medicines were accredited by a pharmacologist. The medicinal mixture was extracted by extracted with 75 % ethanol twice, then infiltration and the resulting ethanol extracts were evaporated and dehydrated under vacuum. The extract powder was weighed (0.585 kg) and used for the experiments by dissolving in pure water or DMEM at the desired concentrations for *in vivo* and *in vitro* studies.

### Ethics statement

All of the study protocols complied with the current ethical considerations of Shanghai University of Traditional Chinese Medicine’s Animal Ethic Committee and the procedural and ethical guidelines of the Chinese Animal Protection Act, which is in accordance with the National Research Council criteria. All animal experiments and procedures were reviewed and approved by the Institutional Animal Care and Use Committee (IACUC) of Shanghai University of Traditional Chinese Medicine and were performed in accordance with the relevant guidelines and regulations.

### In vivo CCl_4_-induced liver fibrosis

Male C57BL/6 mice at 6–8 week (18–20 g) were housed in an air-conditioned room at 25 °C with a 12 h dark/light cycle. The mice received humane care during the study with unlimited access to chow and water. The mice were randomized into two groups: the normal (*n* = 10) and CCl_4_-treated group (*n* = 30). The CCl_4_-treated mice were treated with 10 % CCl_4_ (2 mg/kg of body weight i.p.) diluted in corn oil or with corn oil only (normal) for triweekly and distilled water (by gavage) daily, The CCl_4_-treated mice then divided into CCl_4_-water (CCl_4_, *n* = 20) and CCl_4_-XYXD (XYXD, *n* = 10) from the beginning of first CCl_4_-treatment. At the end of the third week, 10 mice from the CCl_4_-treated group were sacrificed for the fibrosis development assessment. The XYXD treatment group was exposed to the same level of CCl_4_ and administered XYXD at a dose of 0.467 g/100 g body weight, which is equivalent to human doses in clinical therapeutics daily for 6 weeks until sacrifice.

### Hydroxyproline (Hyp) determination

Hepatic hyp content was used as an indirect measure of tissue collagen content. Hyp from liver tissues (50–100 mg) was determined according to the paper we published previously [13].

### In vitro cell culture and treatment

The mouse HSC cell line GFP-Col-HSC was provided by Dr. Ekihiro Seki (School of Medicine, University of California San Diego, CA) and cultured in DMEM with 10 % FBS and 1 % penicillin-streptomycin antibiotics.

XYXD was dissolved with vehicle (DMEM). HSCs were serum starved for 12 h, the GFP-Col-HSCs first treated with XYXD (5, 25 μg/ml) for 1 h, the cells then treated with or without LPS (100 ng/ml) or TGF-β1 (10 ng/ml).

### Reagents

LPS (Sigma; Escherichia coli serotype 055:B5), recombinant human TGF-β1 (R&D Systems) were used in this study. The antibodies used for the western blot analysis, and are p-JNK (catalog no. sc-81502), JNK (catalog no. sc-7345), p38 (catalog no. sc-398305), p-p38 (catalog no. sc-17852-r), p-Smad2 (catalog no. sc-101801), Smad2 (catalog no. sc-39312), p-Smad3 (catalog no. sc-101154), and Smad3 (catalog no. sc-130218), all purchased from Santa Cruz Biotechnology, Inc. NF-κB inducible reporter plasmid were purchased from InvivoGen (cat no: pnifty2-luc, San Diogo, CA). Lipofectamine 2000 transfection regent was purchased from Invitrogen.

### NF-κB luciferase analysis

The GFP-Col-HSC was transfected with the NF-κB inducible reporter plasmid by Lipofectamine 2000 for 12–18 h. The cells were first treated with XYXD (5, 25 μg/ml) for 1 h before treatment with 100 ng/mL LPS or 10 ng/mL TGF-β1. Luciferase activity was measured after 16 h of the treatment with LPS or TGF-β1. Luciferase activity was normalized to the protein concentration of GFP-Col-HSC in each well.

### Measurement GFP-Col-HSC activation

The GFP-Col-HSC normal culture and supplement with XYXD (5, 25 μg/ml) for 36 h. The fluorescent signal HSC was then measured by fluorescent microscopy.

### Quantitative real-time PCR

Total RNA was extracted using TRIzol (Life Technologies, Grand Island, NY), followed by reverse transcription of total RNA to cDNA. cDNA was synthesized using a high-capacity cDNA reverse transcription kit (Applied Biosystems, Foster city, CA). cDNA subsequently underwent quantitative real-time polymerase chain reaction (PCR) using the ABI ViiA™ 7 Dx real-time PCR system (Life Technologies, Grand Island, NY). PCR primer sequences used were used: 18 s rRNA forward 5’-AGTCCCTGCCCTTTGTACACA-3’. 18 s rRNA reverse 5’-CGATCCGAGGGCCTCACTA-3’. Bambi forward 5’- TGAGCAGCATCACAGTAGCA-3’. Bambi reverse 5’- CGCCACTCCAGCTACTTCTT-3’. TIMP1 forward 5’- AGGTGGTCTCGTTGATTCGT-3’. TIMP1 reverse 5’- GTAAGGCCTGTAGCTGTGCC-3’. CCL2 forward 5’- ATTGGGATCATCTTGCTGGT-3’. CCL2 reverse 5’- CCTGCTGTTCACAGTTGCC-3’. CXCL2 forward 5’- TCCAGGTCAGTTAGCCTTGC-3’. CXCL2 reverse 5’- CGGTCAAAAAGTTTGCCTTG-3’. PPAR-γ forward 5’- AACTCCCTCATGGCCATTGA-3’. PPAR-γ reverse 5’- GCATTGTGAGACATCCCCAC-3’. Col 1(α1) forward 5’-TAGGCCATTGTGTATGCAGC-3’. Col 1(α1) reverse 5’-ACATGTTCAGCTTTGTGGACC-3’. α-SMA forward 5’-GTTCAGTGGTGCCTCTGTCA-3’. α-SMA reverse 5’- ACTGGGACGACATGGAAAAG-3’. Gene expression was normalized to 18 s RNA as an internal normal.

### Western blot

Cell samples were prepared in radio immunoprecipitation lysis buffer containing protease inhibitors. After protein quantification, protein samples at 20 μg/lane were subjected to polyacrylamide gel electrophoresis, and then incubated with antibodies for phospho-JNK, JNK, p-p38, p38, p-Smad 2, Smad2, p-Smad 3, Smad 3 with appropriate secondary horseradish peroxidase (HRP)-conjugated antibodies, and developed. Anti-glyceraldehyde 3-phosphate dehydrogenase mouse antibody was purchased from Kangchen and diluted in 1:5000 ratio.

### Immunohistochemistry

The sections were dewaxed in xylene and dehydrated in alcohol. Antigen retrieval was achieved by microwaving in citric saline at 95 °C for 3 min. Thin sections were treated with 3 % hydrogen peroxide for 10 min. The sections were further blocked by 5 % BSA and were then incubated 37 °C with primary antibody against α-SMA (Abcam, UK). The sections were incubated with biotinylated secondary antibody (Boster, Wuhan, China) for 30 min at room temperature. α-SMA expressions were visualized by DAB (Boster, Wuhan, China) staining.

### Statistics

Differences between two groups were compared using the two-tailed unpaired student *t*-test. Differences between multiple groups were compared using one-way ANOVA with a post hoc Dunnett’s test using SPSS 18.0. P values, 0.05 were considered significant. All experiments were performed at least three times and the representative data were presented.

## Results

### Inhibition of CCl_4_-induced liver fibrosis by XYXD

CCl_4_ is known to induce toxicity in the liver by producing highly reactive metabolites, which severely damage hepatocytes and subsequent fibrosis [14]. As shown in Fig 1a, livers of normal mice showed normal lobular architecture with central vein and radiating hepatic cords. After 3 weeks of CCl_4_ treatment, liver centrilobular necrosis, deposition of lipid droplets in hepatocytes, and inflammatory cells infiltration were observed. After 6 weeks CCl_4_ treatment, liver sections revealed collagen deposition, severe fatty changes, whereas, concomitant treatments of XYXD significantly inhibited CCl_4_-induced hepatic damage, as indicated by decreases in hepatocytes degeneration, inflammation, and collagen deposition (Fig 1a).

**Fig. 1:** Effects of Xia-yu-xue decoction (XYXD) on histological changes in CCl_4_-induced liver fibrosis in mice. **a** HE staining (×100), (**b**) Sirius red staining (×100). CCl_4_ (10 %, 2 mg/kg of body weight) was administered intraperitoneally to CCl_4_-treatment mice for tri-weekly and distilled water (by gavage) daily for 6 weeks. The normal mice received an equal amount of corn oil and distilled water (by gavage) daily for 6 weeks. At the end of the third week, 10 CCl_4_-treated mice were for the fibrosis development assessment. The XYXD treatment group was exposed to the same level of CCl_4_ and administered XYXD at a dose of 0.467 g/100 g body weight, which is equivalent to human dose in clinical therapeutics daily for 6 weeks until sacrifice. The number in HE and Sirius red staining was as the same as the animal number in each group

Sirius red staining revealed that mice treated with CCl_4_ for 3 weeks showed prominent red staining in collagen was seen to stretch from portal area to lobular (Fig. 1b). Livers showed marked distortion in architecture, including portal and lobular bridging fibrosis, cirrhotic nodule formation. Collagen fiber percentages in the CCl_4_ groups were significantly decreased in XYXD treated mouse livers.

### HSC activation was inhibited by XYXD in vivo

As sustained deposition of ECM results mainly from HSC activation, α-SMA is a marker of HSCs in hepatic fibrosis [15], and the α-SMA-positive cells are increased gradually in number, mainly located in fibrotic septa following 6 week CCl_4_-treatment. In contrast, a marked reduction of α-SMA-positive HSCs was observed in XYXD liver compared with 6 weeks CCl_4_ liver (6 wk) (Fig 2a).

**Fig. 2:** Effects of XYXD on HSC activation and Col production in CCl_4_-induced liver fibrosis in mice. **a**, liver sections were stained with α-SMA (×200, *n* = 3), Brown staining indicates immunopositivity. **b**, Expression of α-SMA was analyzed using real-time PCR analysis (*n* = 6). **c**, Expression of Col 1(α1) was analyzed using real-time PCR analysis (*n* = 6). **d**, Hyp content of liver tissue was measured. The number in Hyp and Sirius red detection was as the same as the animal number in each group. The data represented the mean ± SD *P < 0.05, * *P < 0.01, *vs* normal mice, ^#^ *P* < 0.05, ^##^ *P* < 0.01, vs 6 wk

The expression of α-SMA in CCl_4_-treated liver samples was also detected by real-time PCR analyses (Fig 2b). The expression of α-SMA and Col 1(α1) increased gradually following CCl_4_ treatment (Fig 2b and c). Compared to 6 weeks CCl_4_ treatment liver (6 wk), XYXD administration resulted in marked reductions in α-SMA and Col 1(α1) (*P* < 0.05). Hepatic hyp content increased in CCl_4_-treated mice gradually, after 3-week CCl_4_ administration, the Hyp content was 206 % of that in the normal group (*P* < 0.05) (Fig 2d). XYXD was found to decrease liver Hyp content significantly (*P* < 0.01).

### The effect of XYXD on HSCs activation in vitro

To reveal the mechanisms responsible for these in vivo observations, we performed *in vitro* studies using GFP-Col-HSC cells, a well-characterized mouse HSC cell line. First, we tested the cytotoxicity of XYXD, as assessed by cell viability. MTT assay showed no significant difference between normal and XYXD treated cells at concentrations 25 μg/ml (data not shown here). Therefore, we used 25 μg/ml of XYXD in subsequent experiments.

### Effects of XYXD on LPS signaling in HSC

We examine whether XYXD inhibits the LPS signaling in HSC. It has been reported that NF-κB activation in HSC is associated with sustained liver inflammation [16]. We investigated the effect of XYXD on NF-κB activity in HSCs. The luciferase array analysis showed that the relative luciferase activity increase significantly 4-fold (*P* < 0.01) with LPS treatment (Fig. 3a) in HSCs. In contrast, treatments at 5 and 25 μg/ml one hour prior to LPS treatment significantly suppressed the LPS-induced NF-κB activation (*P* < 0.05 or 0.01) (Fig 3a). In addition to NF-κB, JNK and MAPK are also activated by LPS in HSC. We therefore examined the effect of XYXD on JNK and MAPK activation. JNK and p38 were quickly phosphorylated in HSC in response to LPS stimulation (Fig 3b). The LPS-mediated JNK and MAPK activation was reduced by XYXD treatment (Fig 3b). We previously reported that Bambi decreased in response to LPS stimulation [11], as expected, LPS treatment increased TIMP1 and decreased Bambi in GFP-Col-HSC cells (Fig 3c) (*P* < 0.05 or 0.01). The XYXD significantly reduced the expression of LPS-induced TIMP1 in HSC (*P* < 0.05 or 0.01). XYXD could inhibit Bambi decrease induced by LPS stimulation (Fig 3c) (*P* < 0.05 or 0.01).

**Fig. 3:** The suppression of LPS-induced signaling by pretreatment of XYXD in HSC. **a**, NF-κB luciferase was measured. One hour after pretreatment with XYXD (5ug/ml and 25 ug/ml), GFP-Col-HSC cells were treated with LPS (100 ng) for 4 h and then transfected NF-κB-luciferase reporter plasmid for 16 h. *P < 0.05, * *P < 0.01, *vs* Un-LPS and No XYXD, ^#^ *P* < 0.05, ^##^ *P* < 0.01, vs LPS and No XYXD. **b**, Western blot analysis for p-JNK, total JNK, p-p38 and total p38. One hour after pretreatment with XYXD (5 μg/ml and 25 μg/ml), GFP-Col-HSC cells were treated with LPS (100 ng) for 30 min. **c**, the mRNA expression of TIMP1 and Bambi was detected by real-time PCR. *P < 0.05, * *P < 0.01, *vs* vehicle, ^#^ *P* < 0.05, ^##^ *P* < 0.01, vs LPS. **d**, the mRNA expression of CCL2 and CXCL2 was detected by real-time PCR. One hour after pretreatment with XYXD (5 μg/ml and 25 μg/ml), GFP-Col-HSC cells were treated with LPS (100 ng) for 4 h. *P < 0.05, * *P < 0.01, *vs* vehicle, ^#^ *P* < 0.05, ^##^ *P* < 0.01, vs LPS. Data represent the mean ± SD of triplicate cultures. A representative result is shown. Similar results were obtained in three independent experiments

Because NF-κB induces an inflammatory response in the liver, we investigated whether XYXD can suppress the induction of inflammatory cytokines in HSC. The pro-inflammatory cytokines of CCL2 and CXCL2 were up-regulated after LPS stimulation (Fig 3d) (*P* < 0.01). The mRNA expression CCL2 and CXCL2 was significantly inhibited by XYXD treatment (Fig 3d) (*P* < 0.05 or 0.01). These results demonstrated that LPS-induced signaling was inhibited by XYXD in HSC.

### Effect of XYXD on TGF-β1 signaling in HSC

TGF-β1 is a classic activator of HSCs and a key mediator in the pathogenesis of liver fibrosis [17]. However, it was rarely reported NF-κB activated in response to TGF-β1 stimulation in HSCs. We assessed NF-κB activity by using the NF-κB luciferase reporter system. TGF-β1 treatment significantly increased NF-κB activity (*P* < 0.01) in HSCs (Fig 4a) (*P* < 0.05 or 0.01). XYXD treatments 1 h prior to TGF-β1 treatment significantly suppressed the TGF-β1-induced NF-κB activation (*P* < 0.05).

**Fig. 4:** Effect of XYXD on TGF-β1-induced signaling in HSC. **a**, NF-κB luciferase was measured. GFP-Col-HSC cells were pretreated with XYXD (5 μg/ml and 25 μg/ml) for 1 h and subsequently treated with TGF-β1 (10 ng/ml) over night, followed by transfect NF-κB-luciferase reporter plasmid for 16 h. *P < 0.05, * *P < 0.01, *vs* Un-TGF-β1 and No XYXD, ^#^ *P* < 0.05, ^##^ *P* < 0.01, vs TGF-β1 and No XYXD. **b**, western blots analysis were analysis for p-Smad2, total smad2, p-smad3, and total Smad3. GFP-Col-HSC cells were pretreated with XYXD (5 μg/ml and 25 μg/ml) for 1 h and subsequently treated with TGF-β1 (10 ng/ml) for 30 min. **c**, the Col1(α1) and TIMP1was measure by real-time PCR. GFP-Col-HSC cells were pretreated with XYXD (5 μg/ml and 25 μg/ml) for 1 h and subsequently treated with TGF-β1 (10 ng/ml) for 24 h. Data represent the mean ± SD of triplicate cultures. *P < 0.05, * *P < 0.01, *vs* vehicle, ^#^ *P* < 0.05, ^##^ *P* < 0.01, vs TGF-β1. A representative result is shown. Similar results were obtained in three independent experiments

The TGF-β1-mediated signaling pathway depends on the phosphorylation of Smad 2/3. As shown in Fig 4b, the protein levels of Smad 2/3 were analyzed. Western blot analysis detected increases in the phosphorylation of Smad 2/3 by TGF-β1, and the inhibition of these increases by XYXD (Fig. 4b). Also, the mRNA expression of Col1 (α1) and TIMP1 significantly increased in response to TGF-β1 stimulation (P < 0.01). XYXD treatment suppress Col1 (α1) and TIMP1 mRNA expression (Fig 4c) (*P* < 0.05 or 0.01). These results indicated that XYXD inhibited TGF-β1-induced HSC activation.

### Effect of XYXD on fibrogenic response induced by LPS plus TGF-β1 in HSC

TGF-β1 treatment increased Col 1(α1) mRNA expression in GFP-Col-HSC cells (Fig. 5), LPS treatment further increased Col 1(α1) mRNA expression in GFP-Col-HSC cells (Fig. 5a) (*P* < 0.05 or 0.01). While, XYXD treatment resulted in dose-dependent decrease in collagen synthesis in GFP-Col-HSC cells (*P* < 0.05 or 0.01). Increased TIMP-1 expression was inhibited by XYXD, with a significantly reduction at the 5 and 25 μg/ml dose level in GFP-Col-HSC cells (Fig 5b) (*P* < 0.05 or 0.01).

**Fig 5:** Effect of XYXD on fibrogenic response induced by LPS plus TGF-β1 in HSC. Col 1(α1) (**a**), TIMP1 (**b**) was measure by real-time PCR analysis. GFP-Col-HSC cells were pretreated with XYXD (5 μg/ml and 25 μg/ml) for 1 h and subsequently treated with LPS for 12 h, then treated with TGF-β1 (10 ng/ml) for 24 h . Data represent the mean ± SD of triplicate cultures. *P < 0.05, * *P < 0.01, *vs* no LPS/TGF-β1, ^#^ *P* < 0.05, ^##^ *P* < 0.01, vs vehicle. A representative result is shown. Similar results were obtained in three independent experiments

### Effect of XYXD on full activated HSC

As shown in Fig 6a, GFP-Col-HSC cell full activated after 36 h culture by measuring GFP fluorescent signal. XYXD treatments at 5 μg/ml and 25 μg/ml suppressed GFP-Col-HSC activation (Fig 6a). The mRNA expression of α-SMA and TIMP1 was decreased significantly by XYXD treatment (Fig 6b and c) (*P* < 0.05 or 0.01). Meanwhile, XYXD increased PPARγ mRNA level compared with vehicle group (Fig 6d) (*P* < 0.01). These results showed that GFP-Col-HSC auto-activated after 36 h culture, and XYXD could inhibit GFP-Col-HSC activation.

**Fig. 6:** The effect of XYXD on full activated HSC. GFP-Col-HSC cells were plated and cultured in 6-well plates for 2 h, then treated with XYXD (5 μg/ml and 25 μg/ml) for 36 h followed by fluorescent microscopy(×100, *n* = 3). Representative pictures are shown (**a**). α-SMA (**b**), TIMP1 (**c**), and PPARγ (**d**) were measure by real-time PCR analysis. The data represented the mean ± SD, ^#^ *P* < 0.05, ^##^ *P* < 0.01, vs vehicle. A representative result is shown. Similar results were obtained in three independent experiments

## Discussion

Xia-yu-xue decoction (XYXD) has used in China for more than 2 thousand years without side effects. However, the anti-fibrotic mechanism of action of XYXD was very limited. In an effect to investigate the inhibitory effect of XYXD on HSC activation, we used (1) CCl_4_-induced liver fibrosis in mice in vivo, and (2) an in vitro model based on GFP-Col-HSC cells treated with or without LPS, TGF-β1 or both. The data demonstrated that XYXD treatment inhibited the accumulation of ECM components in CCl_4_-induced liver fibrosis in vivo. XYXD is capable of inhibiting HSC cellular activated by LPS and TGF-β1 in GFP-Col-HSC lines.

Chronic liver disease commonly leads to liver fibrosis, resulting in development of liver cirrhosis, organ failure, and eventually liver related mortality. Therefore, prevention or treatment of liver fibrosis is the main target in patients with chronic hepatic disorders [18]. Recently, much interest in herbal medicine has been focused on hepato-protective or anti-fibrotic effects. Although lack of strong clinical evidence, many traditional Chinese medicine/recipes/decoctions and drugs such as Yin-chen-hao decoction [13], Xiao-chai-hu decoction (sho-saiko-to in Japan) [19, 20] are used widely in China, Korea, and Japan for thousands of years and reported to have antifibrotic properties. Just like Yin-chen-hao decoction (Inchinko-to in Japan) and Xiao-chai-hu decoction (sho-saiko-to, in Japan), Xia-yu-xue decoction first described in Shanghan Lun, while, there were rare limited information about the anti-fibrotic effects of XYXD. So it is very urgent to investigate the mechanism of action of XYXD. In this study, we found XYXD inhibit α-SMA and Col 1(α1) expression, which indicating HSC activation were suppressed in CCl_4_-induced liver fibrosis in vivo.

LPS levels increase in the systemic circulation owing to changes in the intestinal mucosal permeability after liver injury [21, 22]. LPS plays a key role in hepatic fibrogenesis by enhancing HSC activation [23]. NF-κB activated in response to LPS-mediated TLR4 activation [24]. So we want to know whether XYXD inhibit LPS signaling through NF-κB. In the present study, NF-κB luciferase increased in response to LPS stimulation and was inhibited significantly by XYXD treatment. Our study also demonstrated that XYXD suppressed both JNK and p38 signaling pathways induced by LPS. Furthermore, we approved that the mRNA expression of CCL2 and CXCL2 was also suppressed by pretreatment with XYXD.

In response to liver injury, HSCs undergo activation process and produce ECM [25]. The process is primed by various growth factors, where TGF-β1 is the most important profibrogenic mediator. It was well reported the pro-inflammatory cytokine through NF-κB enhance TGF-β1 signaling [1, 23]. However, whether TGF-β1 could induce NF-κB activation was largely unknown. Our results showed that NF-κB activity increased almost 2-fold in response to TGF-β1 stimulation, and XYXD could inhibit NF-κB activity induced by TGF-β1. Moreover, the signaling pathway activated by TGF-β1 involves phosphorylations of Smad 2 and Smad 3 [26, 27], which were also inhibited by XYXD. These data suggest that XYXD blocks fibrogenesis as mediated by TGF-β1 signaling pathways.

We used LPS plus TGF-β1 to mimics the complex environment in vivo. The mRNA expression of Col 1(α1) and TIMP1 increased significantly using LPS plus TGF-β1 stimulation compared with TGF-β1 alone in GFP-Col-HSC cell line. However, XYXD treatment decreased the enhancement of TGF-β1 plus LPS-induced Col 1(α1) and TIMP1 mRNA expression. This may be due to the inhibitory effect of XYXD on NF-κB and TGF-β1 signaling, and the further mechanism should be studies in future research.

## Conclusions

This study demonstrated that XYXD reduce HSC activation in CCl_4_-induced liver fibrosis in mice. The inhibitory effects of XYXD on HSC activation may be caused, at least in part, by suppressing on NF-κB and TGF-β1 signaling pathway.

## Abbreviations

α-SMA: Smooth muscle actin alpha
CCl_4_: Carbon tetrachloride
CCL2: Chemokine (C-C motif) ligand 2
CXCL2: Chemokine (C-X-C motif) ligand 2
HSC: Hepatic stellate cell
Hyp: Hydroxyproline
LPS: Lipopolysaccharide
NF-κB: Nuclear factor-κB
TGF-β1: Transforming growth factor
TIMP1: Tissue inhibitor of metalloproteinases
XYXD: Xia-yu-xue decoction
